The article "Visual Evaluation of Urban Streetscape Design Supported by Multisource Data and Deep Learning" was retracted in 2023. Reasons: unreliable results or conclusions; concerns about the data; concerns about the peer review; concerns about the citations.

# Visual Evaluation of Urban Streetscape Design Supported by Multisource Data and Deep Learning

**DOI:** 10.1155/2022/3287117

**Published:** 2022-02-07

**Authors:** Guanqing Feng, Guangtian Zou, Pengjin Wang

**Affiliations:** ^1^Department of Architecture, Faculty of Architecture, Harbin Institute of Technology, Harbin 150006, Heilongjiang, China; ^2^Key Laboratory of Cold Region Urban and Rural Human Settlement Environment Science and Technology, Ministry of Industry and Information Technology (Harbin Institute of Technology), Harbin 150006, Heilongjiang, China; ^3^Department of Landscape Architecture, Faculty of Horticulture and Landscape Architecture, Northeast Agricultural University, Harbin 150030, Heilongjiang, China

## Abstract

This paper integrates classical design theory, multisource urban data, and deep learning to explore an accurate analytical framework in a new data environment, providing a scientific analysis path for the “where” and “how” of greenways in a high-density built environment. The analysis is based on street view data and location service data. Through the integration of multiple data sources such as street scape data, location service data, point-of-interest data, structured web data, and refined built environment data, a systematic measurement of the key elements of density, diversity, design, accessibility to destinations, and distance to transport facilities as defined in the Five Elements of High Quality Built Environment (5D) theory is achieved. The assessment of alignment potential was carried out. The key factors influencing the aesthetics of the street were identified. Based on an extensive landscape perception-based survey, it was found that although different respondents had different views and preferences for the same street scape, their preferences were overwhelmingly influenced by the visual quality of the street scape aesthetics itself, with higher aesthetic quality of the landscape.

## 1. Introduction

In the landscape engineering system, landscape resources are divided into 3 categories: human resources, natural resources, and landscape visual resources [1]. Of these, how to evaluate landscape resources, especially landscape aesthetics, has not yet been agreed upon by the landscape community and is expressed in practice in inconsistent ways [2]. Most people will own their own opinions on whether a particular landscape is aesthetically significant, and there is an increasing emphasis on the role that everyday landscapes play in everyday life [3]. In the case of landscape aesthetics, there are many controversies in the industry. Often, the ambiguity of landscape aesthetics is due to the subjectivity of its definition, the lack of standardisation of its methodology, the lack of clarity in its practical application, and its own particular lack of replicability [4]. In contrast, it has become increasingly evident in the last decades that the visual aesthetic quality of landscapes is considered an important resource for the maintenance of people's psychological well-being, as well as for the conservation of biodiversity, cultural heritage, and the potential of landscapes [5–8]. Therefore, the development of a methodology for the analysis and evaluation of landscape aesthetics that can be accepted by the scientific community as a whole is a major challenge facing the academic community today.

The visual aesthetic quality can be viewed from the same 2 perspectives. From an objective point of view, the visual aesthetic quality of a landscape is determined by the elements it contains and its properties. The subjective point of view, on the other hand, explores the status of the visual aesthetics of the landscape within people and the subjective feelings it brings to them, starting from their subjective inner thoughts. Paper [9] has also proposed in the systematisation of landscape engineering that the intentional content of the landscape carries objective factors and the real content of the landscape carries subjective factors and that the aesthetic feeling of the landscape always contains these 2 types of basic components, while the controlling role is played by the intentional content of the landscape. Based on the above background, two approaches to assessing the visual aesthetics of landscapes are commonly used in the industry [10].

In addition, certain specific visual attributes of the landscape are also considered important, such as openness, consistency, colour contrast within space, vividness, and a sense of nature [11]. In terms of living and architecture, elements such as traditional architectural style, family house style, architectural details, and the overall living environment were most often preferred by occupants [12–15]. With regard to the subjective characteristics of respondents, industry studies have demonstrated that factors that contribute significantly to and influence people's visual aesthetic preferences for landscapes include occupation, education level, and gender [13].

With the gradual development of the new data environment, multidimensional exploration of the built environment at a finer scale across the country has become possible, advancing the need for more refined quantitative research on urban design. On the one hand, new analysis techniques are emerging, and the gradual application of GIS technology and Geodesign concepts in the field of urban design provides quantitative analysis tools, and spatial analysis supported by intelligent algorithms is expected to provide scientific support for spatial background identification and line selection effectiveness assessment. On the other hand, the emergence of high-precision open data such as road networks, points of interest, and building base maps provides new opportunities for the measurement of traditional unmeasurable data [16], and user profiles supported by multiple sources of data can also help to target accurate design. These new data and technologies can provide refined spatial feature extraction on the human scale, thus measuring various spatial quality that was previously difficult to assess accurately and offering new possibilities for human-centred urban design [17]. In this context, quantitative analysis of 5D elements, which were previously difficult to apply effectively in practice, has also emerged [18]. For example, location-based service (LBS) location data can be used in comparison to traditional measurement methods. Location-based service (LBS) location data can provide information on the behavioural activities of people over a wide range of time periods [19, 20]; street view images (SVIs) can be combined with machine learning; green visibility and street scape quality can be evaluated more efficiently and finely [21]; the combination of street base data and spatial design network analysis (sDNA) software enables large-scale and accurate street network accessibility measurements [22].

In summary, the rapid emergence of multisource urban data offers the possibility of in-depth analysis using the 5D concept to measure the quality of the built environment. Most of the existing studies focus on a single dimension of built environment quality, while only a few researchers have combined two or more dimensions to measure street quality [23], and systematic analyses that integrate the five elements of the built environment at once are rare. In response to this research situation, this study aims to make use of new data and technologies to systematically measure many elements of street quality from a user-centred perspective and to compensate for the lack of scale and accuracy in traditional quantitative analysis.

## 2. Related Work

Although the scope of landscape visual evaluation has covered many aspects, most studies and cases in the past have been on large-scale natural landscapes; for example, some scholars have used example-validated methods such as psychological and psychological preferences to establish mathematical models for visual quantitative analysis and make a comprehensive evaluation of tourism resources from the perspective of visual aesthetics [24]. In recent years, the focus of foreign research on visual evaluation of landscapes has gradually shifted from the development of natural areas to the evaluation of urban and suburban areas, using visual evaluation methods to guide the planning and construction of cities. Especially after entering the 21st century, with the application of new technologies such as geographic information technology and computer image processing technology, the visual research and application of urban landscape, which was previously not easy to carry out due to the composition and influencing factors of urban landscape being too complex, has also developed greatly [25].

In the 1960s, some Japanese scholars explored the construction of greenery in the street space environment, and it was found that the green colour of plants can stimulate the human brain through vision; i.e., there is an obvious correlation between people's evaluation of their feelings about the street and the street environment they are in [26]; through the study of the “Report on the Basic Survey of Greenery in Suginami District,” it was confirmed that green vegetation can improve the satisfaction of the landscape in residential areas, and at the same time it also helps people to identify the landscape; countries such as Europe and the United States have also suggested that the amount of vegetation present in the visual field in large quantities contributes to the reporting of landscape evaluation. These research results are also gradually being recognised internationally, and a large number of scholars are beginning to experiment with and provide advice on the visual evaluation of landscapes in roads, parks, and residential areas, in order to improve the visual quality of landscapes in residential environments [27, 28].

In 1990, some scholars in China began to introduce theories related to visual evaluation from abroad, which laid a preliminary theoretical foundation for the development of visual landscape in China. In the same period, some scholars began to make preliminary explorations of examples in the evaluation of the visual environment of the landscape, for example, the exploration of landscape resource management and visual impact assessment methods; from urban design theory, the basis was chosen to select impact factors to conduct research on the control of the visual environment of urban landscapes [29]. This also includes a large number of evaluations of the visual environment of landscapes relating to urban streets, such as the use of multifactor evaluation method to evaluate the visual landscape of roads; through multifactor evaluation method as well as questionnaire survey method to evaluate the visual landscape of urban roads; exploration of the applicability of urban road visual analysis; the use of landscape comprehensive evaluation index method to evaluate the quality of the landscape visual environment of Hong'an County Yingbin Avenue; the index of the visual evaluation of street landscape is divided into horizontal interface (street surface) and vertical interface (the three factors of street scape visual evaluation are divided into horizontal interface (street level), vertical interface (buildings, street trees), and street facilities); the visual index and SD method are proposed and applied to investigate urban streets, so as to obtain people's comprehensive evaluation of the visual environment of streets; two subjective evaluation methods, namely, the cognitive map method and the psychological evaluation method, are used to conduct field research on a number of living streets in Chongqing in the form of questionnaires, so as to derive the physical environment characteristics of street aesthetics.

In addition, modern information technology has also been widely used in the evaluation of the visual environment of the landscape at this stage in China, for example, the use of virtual reality technology and panoramic holographic technology to recreate the landscape along the Yellow Crane Tower in three dimensions, making the landscape simulation more in line with people's visual habits; the use of 3S technology to quantitatively evaluate the possible visual impact of new railways [30]; the use of Arc GIS visual field analysis function to analyse the visual field characteristics of the trails in the National Forest Park of Liaoning Province; the comprehensive evaluation of the aesthetic quality of Hangzhou Garden from the perspective of the public; the identification of green plant areas from Google Street View photos and the calculation of “green visual quality” at street scale. The study identifies areas of greenery from Google Street View photos, calculates a “green visual index” on the street scale, and suggests that street view photos could be of great use in future urban environmental planning. In general, the assessment methods and techniques used are constantly being developed and updated, and the objects and content of the assessment have been greatly expanded and deepened.

## 3. Study Site and Methodology

### 3.1. Study Site

The Shanghai area was chosen as the study site because local data was easily available and the area is known to be a multicultural gathering place where different cultures merge and are very prominent in reflecting the visual aesthetic preferences of different groups in the streetscape. With a planned area of 220 *km*^2^, the area is positioned as a regional leader in opening up to the outside world and economic development, a base for high-tech industries, and a new modern urban area of high standard. Over the past 30 years, the urban space has developed from the north-east to the south-west, with the eastern part of the city being the birthplace of the development of the entire development zone [31]. The area of green space in the area has become more and more concentrated due to the needs of the development of the region, in contrast to the increasingly convenient transportation, the development of housing and public buildings, and the development of various industries.

### 3.2. Research Methodology

As mentioned earlier, one of the focuses of this study is to focus on the visual aesthetic preferences of fire-escapes at the subjective level. Therefore, subjective opinions from different groups of people had to be collected in order to determine local preferences for the visual aesthetics of the streets. Because opinions are open-ended and influenced by the personal preferences of the participants, this objective can best be achieved through the interview method of the qualitative research process [32]. And in landscape studies, extracting participants' perceptions through images has become a staple of the industry; this has proven to be an effective method. Building on this, Yohan Shao proposed that a subjective interview method using photographs as a basis is more effective in gathering opinions about the landscape [26]. Therefore, this study uses the experiential landscape annotation method in conjunction with the photo-oriented interview process and the basic principles of pinpoint notation to collect valid data for the study and analysis of the visual aesthetics of stroboscopes [28].

Firstly, the study area was set up along the main regional roads as reflected in the urban development map, with the route maintaining a good sense of spatial continuity, and the interviewing population would travel through the corresponding streets and record the characteristics of the visual experience of the street as perceived at each location. It is important to note that what is recorded are the more salient features at that location and not just the features that can be seen in the photographs, but also the psychological features etc. The photographs we use are simply a means of recording location and sequence (Figures 1 and 2).

These findings were then recorded in a table to clarify the quality of the different dimensions of visual aesthetics and the reasons for them. As the aim of this paper is to identify and assess the visual aesthetics of streets in urban areas, it was necessary for the participants to have some knowledge of the local area and therefore only local residents were selected for the data sampling. Local participants were selected from a mix of local construction and planning related professionals and nonprofessional local residents, a total of 90 people. It was also ensured that the participants covered three groups: older, middle-aged, and younger. The reason for this is that the different age groups have different insights into the local area and their interaction with the local environment, as shown in Figure 2.

In this study, the interviews were selected to be conducted at the regional site, in conjunction with a field visit survey. This method also proved to be interactive and effective in reducing the length of the interview, thereby reducing the resources required for the study [29]. Each set of interviews lasted between 40 min and 1 h, depending on the speed of the participant's choice and the details of the interview.

## 4. Study Design

### 4.1. Analytical Framework and Key Indicators

The study consisted of 4 main research steps: data collection, key feature extraction, alignment potential assessment, and feature mapping (Figure 3). Firstly, the study collected data from multiple sources such as LBS, POI, road network base data, MMT business hours data, SVIs, and refined built environment data for both sides of the Suzhou River area. Secondly, eight key variables representing the 5D theory were extracted from the dataset. In addition, as this is an implementation-oriented project, the maximum continuous nonmotorised section width of the road section is also used as a constructible indicator. Again, the relative weight of each of the nine factors in the six dimensions was calculated using AHP hierarchical analysis, and the indicators were then integrated to form an overall greenway suitability score. Finally, a radar map is used to draw a characteristic picture of a typical road section. The integrated multidimensional analysis can provide accurate guidance for the selection of greenway alignments and section design.

### 4.2. Study Case: Suzhou River Area, Shanghai

The study area covers the southern part of the Jing'an District on both sides of the Suzhou River, from North Henan Road in the east to Jiangning Road in the west, from West Beijing Road in the south to Jiaotong Road in the north, with a total land area of approximately 440 h *m*^2^. The Jing'an District is small in area and has a high population density of approximately 64,000 people/ *km*^2^, ranking first among all districts in Shanghai. However, at the end of 2016, the per capita parkland area in Jing'an was 2.7 *m*^2^ /person, the third lowest in the central city, as shown in Figure 4. At the same time, the area has limited space for additional green space as there is less land available for construction [22]. Therefore, a study on the construction of urban greenways in this area can help to address the problems of environmental degradation and spatial disorder caused by high-density urban development and construction [23].

The activity density measurement was carried out based on Tencent's LBs location service data, and six representative time periods were selected on weekdays and weekends to capture the real-time crowd location distribution using Python computer language. A total of 20,405 data points were collected on weekdays and 15,436 data points were collected on weekends. As showed in Figure 5, each point represents a grid of 30 m in size, with high and low values representing the intensity of activity. The data were then preprocessed using ArcGIS for cleaning, spatial alignment, and kernel density analysis, and a spatial merging tool was used to translate the LBS into street segments with a 50 m buffer to reflect the current intensity of use in and around the street. This study shows that the buffer zone is a good reflection of the built environment characteristics of Shanghai.

For the street pedestrian count, a new method proposed by researchers from the City University of Hong Kong, Beijing Jiaotong University, and Tongji University was used, which showed good agreement with the field manual observation data in an empirical study in Tianjin (Figure 5). In this study, we firstly generated street scape sampling points with a sampling spacing of 30 m and calculated the latitude and longitude of each sampling point as well as the geographic orientation of the street segment where the sampling point was located; secondly, we set the street scape download parameters and obtained multiple phases of street scape for the sampling points in 2018–2019 by calling the APIs of Baidu and Tencent Street View [2]; then we cropped the street scape to cover only the pedestrian area on the left and right sides of the street as much as possible; finally, the LDCF algorithm is used to detect pedestrians. In addition, since the street view obtains the number of pedestrians at a certain point in time, and there are multiple sampling points in each street segment, and pedestrians are constantly moving in space and time, the average value of sampling points in each street segment is used instead of the pedestrian count in that street segment.

Diversity is measured in 2 ways, functional diversity based on POI data and average daily business hours based on Meituan data. With the popularity of mobile Internet, the increasing correlation between online data and physical facilities makes this data source an important resource for urban research. The study used Python and the Gaode Map API to extract 2,189 POIs in the study area, all of which were classified into different categories including food and beverage services, education, medical services, and transportation facilities, which can form a spatial distribution feature of various functional facilities (commercial, business, food and beverage, public services, etc.) in the city (Figure 6).

Once the data were obtained, functional diversity values were measured in 2 steps: (1) calculating the total number of POIs for each unit within a daily walking distance of 15 min and 1,000 m [25]; (2) measuring diversity using the widely used entropy index [26], which has been applied in many built environment studies [13], calculated as

(1) $$\begin{array}{c} D_{i}=-\sum_{i=1}^{R}p_{i}\times \;\ln\;p_{i}, \end{array}$$

where *p*_*i*_ is the proportion of the total number of POI types in a street unit, *R* is the total number of main functional categories, and the diversity value (*D*_*i*_) is between 0 and 1. The greater the diversity index for each street unit, the better the mix of facilities. Average daily hours of operation based on Meituan data can reflect the economic vitality of the street. Since the hours of operation vary greatly from business to business, the hours of operation of shops are categorised as 06:00 am to 15:00 pm, 09:00–10:00 am to 15:00–18:00 pm, and 08:00–10:00 am to 18:00 pm: 00–10:00 am to 18:00–21:00 pm, 09:00–10:00 am to 21:00–22:00 pm, 06:00 am to 22:00 pm–0:00, 06:00 am to 0:00–03:00 am, 11:00–12:00 pm to 03:00–06:00 pm, 24 hours of operation in 8 categories (Figure 7). The shop hours were then aggregated to nearby streets to compare the overall hours of operation for each street.

## 5. Analysis of the Results

### 5.1. Results of the Analysis of Key Dimensions

For comparison purpose, the calculated results for the 9 subitems of the 6 dimensions related to urban greenway suitability were sorted into 5 categories from highest to lowest value, based on the ArcGIS quantile method.  Figure 8 shows the scores for the eight variables from the five elements of the built environment in the study area, which measure the potential of each road section as an urban greenway alignment. In general, sections with higher development intensity and vibrancy are also more attractive to people and should be prioritised for inclusion in the slow-moving space system (Figure 8(a)). At the same time, streets with high functional diversity and longer operating hours offer a richer range of activities (Figure 8(b)). In addition, a higher quality of street space is physically and emotionally pleasing and can enhance the attractiveness of the street, making it more suitable for inclusion in the planned system of slow-moving space. There is no clear pattern in the intensity of development zones on the streets within the study area, and there are significant differences between road sections (Figure 8(c)). Considering the huge pulling effect of metro stations and the influence of pedestrian accessibility on pedestrian flow, priority should also be given to selecting streets with high scores on these two indicators when shaping the slow walking space system, which will help to improve the accessibility of the whole slow walking space system (Figure 8(d)).

Finally, the wider the nonmotorised road section width, the more likely it is to become a slow potential space under certain conditions. As shown in Figure 9, in the study area, the maximum continuous nonmotorised space is wider in sections such as Hengfeng Road, Hengtong Road, and Guangfu Road near the Hanzhong Road metro station on the north bank of Suzhou River, Qufu Road, North Xizang Road, Jinyuan Road, and Wuzhen Road near the Qufu Road metro station, and Xinzha Road on the south bank of Suzhou River. Priority should be given to the inclusion of the slow-moving space system.

### 5.2. Weight Determination Based on Hierarchical Analysis

By inviting more than 10 experts in the fields of architecture, planning, and landscape to conduct a comparison using the hierarchical analysis and evaluation method (AHP), the weight of the above-mentioned factors influencing the evaluation of the potential of urban greenway alignment was calculated. Based on the aforementioned analysis, nine factors in six dimensions were selected to build the indicator layer, and the importance of the indicators was compared by means of a two-by-two discriminant matrix, with the importance levels assigned on a scale of 1 to 9, with higher values indicating a higher importance of the former than the latter.

### 5.3. Greenway Alignment Potential Assessment

Street data for a total of 9 indicators in 6 categories were further standardised so that the results were mapped to a range of values from 1 to 5, making the indicators comparable, and weighted and aggregated according to the weights of the elements determined by AHP above.

(2) $$\begin{array}{c} \text{Potential value}=\sum_{i=1}^{9}D_{i}\times X_{i}, \end{array}$$

where *D*_*i*_ are the influencing factors for each category of alignment potential from Table 1, and *X*_*i*_ are the corresponding weights.

On this basis, a comprehensive potential value for the urban greenway network can be calculated, the degree of which can be divided into five categories from high to low, arranged dark green to light green (Figure 10). The sections of Hengfeng Road, Hengtong Road, and Hanzhong Road near the Hanzhong Road Station on the north side of the Suzhou River, the Qipu Road Garment Wholesale Market at the Qufu Road Station, and the sections of Xinzha Road, Taixing Road, and Wuding Road on the west side of Wuding Road Street have high potential values for greenway construction, are coherent and have the potential to form vertical links with the Suzhou River, and have a higher degree of urgency for the construction of a slow-moving network, and should be given priority consideration for inclusion in the greenway planning system.

### 5.4. Characterisation of Road Sections with New Data and Technology

This digital analysis model is used not only to assess the potential for route selection, but also to quickly generate a comprehensive profile of each section. It provides a scientific and systematic characterisation of the “how” of the greenway in a high-density built environment and allows for the subsequent design of each section to be targeted and to show the corresponding guiding strategies of human-scale characteristics.

Two of the more noteworthy categories in the aforementioned urban greenway potential assessment are presented here as case studies. The first category is the streets with the highest potential for greenway construction, such as Meiyuan Road (the section between Tianmu Xi Road and Republican Road, Figure 11), which has taller buildings and high development intensity on both sides, a commercial type of building interface on both sides of the street, close proximity to the metro station Qufu Road Station, better spatial background conditions, narrower red lines, and nonmotorised widths, but wider pedestrian access, strong pedestrian accessibility, and suitability for slow walking. The spatial use vitality is high, with high activity, street vitality, and economic vitality, and a low distribution of flows in the current and planned context. Spatial perception of street quality is high, with a high level of green views, and street space enclosure is high, while pedestrian visibility is slightly lower.

The spatial context is good, with a high intensity of development and accessibility to public transport, but the proximity of green spaces and water bodies is poor and the accessibility to everyday life is poor. Overall, the spatial base is good, the spatial use is dynamic, the perceived quality of the space and the environment is excellent, and it only requires microrenewal at street level to improve its pedestrian accessibility and can be incorporated directly into the greenway planning system.

## 6. Conclusions

The analysis technique proposed in this study still has some limitations. Firstly, the current analysis is mainly applicable to the assessment of greenway alignment potential and road segment characteristics, but not for large-scale greenway selection, which needs to be explored in further research. Secondly, the reliability and validity of multiple Internet data, such as LBS and POI data, can be further improved. Future research can further integrate data from multiple sources for calibration in order to improve the accuracy. In addition, the pretrained deep learning model used in this study is unable to distinguish specific types of green vegetation by the spatial features of plants in street scape images.

## Figures and Tables

**Figure 1:** Selected photographic records of participants.

**Figure 2:** Photographs of some elements affecting visual perception.

**Figure 3:** Research design framework.

**Figure 4:** Scope of the study.

**Figure 5:** Example of street pedestrian count extraction.

**Figure 6:** POI extraction example.

**Figure 7:** Example of street business hours distribution extraction.

**Figure 8:** Distribution of the 8 categories of factors influencing the potential for greenway alignments.

**Figure 9:** Distribution of nonmotorised section widths.

**Figure 10:** Distribution of potential values for the construction of urban greenways.

**Figure 11:** Characterisation of high potential sections of urban greenway construction.

**Table 1:** Assessment of urban greenway potential: impact weights for 6 dimensions and 9 subdimensions.

Key dimensions	Subitem	Weight (%)
Density	Activity density	10
	Pedestrian density	10
	Building density	5
Diversity	Functional diversity	15
	Business hours	20
Design	Visual quality	10
Distance between transportation facilities	Distance from subway	10
Destination accessibility	Section accessibility	10
Constructability	Continuous nonmotorised section width	10

## Data Availability

The dataset used in this paper is available from the corresponding author upon request.
